# Effects of *Descurainia sophia* on Oxidative Stress Markers and Thirst Alleviation in Hemodialysis Patients: A Randomized Double-Blinded Placebo-Controlled Cross-Over Clinical Trial

**DOI:** 10.1155/2022/2001441

**Published:** 2022-11-04

**Authors:** Masoumeh Asgharpour, Noora Enayati, Mohammad Rezaei Sadrabadi, Mana Mohamadi Afrakati, Armin Khavandegar, Parham Mardi, Amirhesam Alirezaei, Ali Taherinia, Mahmood Bakhtiyari

**Affiliations:** ^1^Department of Nephrology, Rouhani Hospital, Babol University of Medical Sciences, Babol, Iran; ^2^Department of Phytochemistry, Medicinal Plants and Drug Research Institute, Shahid Beheshti University, Tehran, Iran; ^3^Department of Internal Medicine, Shahid Beheshti University of Medical Sciences, Tehran, Iran; ^4^Department of Internal Medicine, Emam Ali Hospital, Alborz University of Medical Sciences, Tehran, Iran; ^5^Student Research Committee, Alborz University of Medical Sciences, Karaj, Iran; ^6^Clinical Research and Development Center, Shahid Modarres Hospital, Department of Nephrology, Shahid Beheshti University of Medical Sciences, Tehran, Iran; ^7^Department of Emergency Medicine, Alborz University of Medical Sciences, Karaj, Iran; ^8^Non-Communicable Diseases Research Center, Alborz University of Medical Sciences, Karaj, Iran; ^9^Department of Community Medicine, School of Medicine, Alborz University of Medical Sciences, Karaj, Iran

## Abstract

**Background:**

Patients undergoing hemodialysis (HD) are regularly exposed to oxidative stress and inflammation and may suffer from thirst distress with no definitive treatment to address these complications. *Descurainia sophia* (DS) has been used to alleviate thirst in traditional Persian medicine. This study aimed to assess the effectiveness of DS on oxidation factors and thirst score in HD patients.

**Methods:**

This study was conducted on fifty-three HD patients referred to Tehran Shahid Modarres hospital. The patients were randomly divided into two groups: Group 1 received DS for six weeks, then underwent four weeks of washout period followed by six weeks of placebo treatment, while group 2 received placebo initially followed by treatment with DS. Biochemistry, malondialdehyde (MDA), and total antioxidant capacity (TAC) were measured in four phases: at the beginning, before washout, after washout, and at the end of the study. The patient's body weight was recorded at the start of each session to assess interdialytic weight gain. Thirst scores also were measured using a visual analog scale.

**Results:**

A total of 53 patients, including 23 (43.4%) male and 30 (56.6%) female subjects, were included in the study. The results showed a reduction in thirst score (*p*=0.001), cholesterol levels (*p*=0.046), triglycerides (0.003), and MDA (*p* < 0.001) following the four-week administration of DS treatment in HD patients. The mean levels of TAC were increased (*p* < 0.001), and calcium, as well as Na+, remained unchanged (*p* > 0.05). Also, a significant decrease in the patient's weight was observed (*p* value <0.001). This effect persisted after shifting to a placebo. However, the two groups had no significant difference (*p* value = 0.539).

**Conclusion:**

DS powder-mixed syrup may benefit HD patients by facilitating free radical scavenging and alleviating thirst distress with minimal adverse effects. The seeds could therefore be utilized as a complementary therapy for hemodialysis patients.

## 1. Introduction

Adherence to restricted liquid intake is crucial to prevent chronic volume overload and cardiovascular complications in hemodialysis patients. Restraining fluid consumption is also used to maintain normovolemia in end-stage renal disease (ESRD) patients; however, fluid restriction is associated with thirst distress, which may conversely lead to large interdialytic weight gain [1]. Thirst sensation is regulated by central osmoreceptors, which respond to plasma volume and osmolarity through arginine-vasopressin hormone. Therefore, several factors, including sodium intake, volume sensors, renin-angiotensin system, blood urea levels, and even psychological factors, are linked to thirst distress. As a common finding in patients undergoing dialysis, xerostomia elicits the need for fluid intake and subsequently results in chronic volume overload [2, 3]. This reciprocal phenomenon would lead to unfavorable outcomes and diminished life quality in this subset of patients. The precise mechanisms of thirst distress are unclear, and no potential thirst-suppressant drugs have been developed [2–11].

Complementary and alternative medicine (CAM) is a promising accessory treatment for chronic diseases, including patients undergoing hemodialysis. Herbal remedies are frequently used, amongst other CAM methods [12]. Topical application of eugenol nanoemulsion in HD patients on pain control [12] and effect of hydroalcoholic extract of *Allium noeanum* Reut. ex Regel on decreasing renal stone and creatinine [13] are examples of herbal remedies in CAM treatment and effect of reflexology and Swedish massage on restless legs syndrome and sleep quality [14], and effect of foot reflexology on the quality of sexual life in hemodialysis patients [15] are examples of nonherbal remedies in CAM treatment.

In traditional Persian medicine (TPM), seeds of *Descurainia sophia* (DS), commonly known as fixweed, herb Sophia, tansy mustard, and Khak-e-sheer in Iranian traditional medicine [16], are considered a thirst-quencher remedy. The herb grows in several parts of the world with yellow flower petals and an average length of about 80 centimeters. A considerable body of the literature has reported a broad spectrum of therapeutic usage [17–29] for the herb, including free radical scavenging [18], antiparasitic [19], antidiarrheal [20], anti-inflammatory, antioxidant [21], anthelmintic, analgesic, antipyretic [22–24], oncocidal [25], antiarrhythmic [26], stool softening [27], and asthma preventing properties of DS seeds [28]. In a study conducted by Pourmasoume et al., consumption of DS for four months was a suitable therapy for alleviating IBS-C symptoms and could be a beneficial option for first-line treatment [29]. Furthermore, DS showed a significant protective effect against gentamicin-induced acute kidney injury by alleviating biochemical and histological markers of renal toxicity in male rats [16].

By isolating and extracting the chemical components of DS in previous studies, 15 free and protein amino acids were identified, with glutamic acid being the most frequent free amino acid [28]. Studies have also noticed that DS is a rich source of polyunsaturated fatty acids and have identified at least ten specific fatty acids, although with discrepancies in the proportion of each compound. A report demonstrated that linoleic acid comprises the greatest proportion of the fatty acid (40%) [17], whereas another study has reported palmitic acid as the major component (27.45%) [18]. It is worth noting that 15 steroidal compounds were also identified [28].

DS seed extracts are reported to have 15 distinct flavonoid components and seven coumarin derivatives. The presence of flavonoids such as kaempferol-hexoside, *β*-amyrine, isorhamnetin, serotonin, herbal cholesterol (ergosterol), quercetin, morin, and *β*-sitosterol; and coumarins including namely scopoletin, scopoline, isoscopoline, xanthtoxol, xanthotoxin, psoralene, and bergapten in DS seed extract has been confirmed in previous studies [28, 30–32]. Moreover, other constituents identified by using gas-chromatography mass spectroscopy consist of menthol (11.27%) and cis-*β*-ocimene (20.1%). Previous experimental studies revealed that consuming up to 2400 mg/kg of SD is safe and well-tolerated with no adverse effects, while in the current study, relatively lower doses were administered [16]. Moreover, the clinical studies did not indicate any significant adverse effects of DS, demonstrating that it is a safe herbal medicine.

The anti-inflammatory and antioxidant effects of DS have been proven in previous experimental studies [24, 33]. Mirzaei et al. showed antioxidant effects of this herb in vitro [21]. They suggested that DS's antioxidant effect is due to free radical scavenging [24]. These effects may lead to the alleviation of thirst distress.

This study aims to identify the impact of DS consumption on certain blood biochemical indices, thirst, interdialytic weight gain (IDWG), serum inflammatory markers, and lipid peroxidation status in hemodialysis patients through a cross-over trial design.

## 2. Methods

### 2.1. Study Design and Samples

This double-blinded randomized cross-over clinical trial was carried out at Tehran Shahid Modarres hospital, Shahid Beheshti University of Medical Sciences and Health Services, in 2018. The study design and objectives were fully elaborated for each patient. Written consent acknowledging willing participation was obtained for each patient.

This study adhered precisely to the ethical principles of the World Medical Association Declaration of Helsinki, and all procedures were validated by the Ethical Committee of Research at Shahid Beheshti University of Medical Sciences (IR.SBMU.RETECH.REC.1397.299). This work was registered in the Iranian registry of clinical trials. Trial registration number: https://clinicaltrials.gov/ct2/show/IRCT20170725035305N3.

Of the sixty-two participants screened for eligibility, nine patients were excluded/removed from analysis due to the following reasons: hospital admission for pneumonia (*n* = 2), kidney transplantation (*n* = 1), catheter-related infections (*n* = 2), nonadherence to study protocol (*n* = 2), death during the trial (*n* = 1), myocardial infarction (*n* = 1), and other exclusion criteria. The primary analysis was conducted on the data derived from the remaining 53 patients in the study.

Subjects met inclusion criteria if they were 18–70 years old, on hemodialysis for more than three months KT/V > 1.2, were insensitive to *D. sophia* or any herbal remedy, and had no history of active infection in the past month using AVF for hemodialysis. Patients were excluded if they were sensitive to *D. sophia* or any herbal remedy, had a history of active infection in the past month, or were unwilling to participate for any reason, or to use permcath or AVG for hemodialysis, or hospital admission for any reason in the past month and during the study period. Prescriptions regarding dialysis and the dialyzer itself were similar among the participants. Conventional drugs were continued for each patient till two weeks before the initiation of the study, when all anti-inflammatory medications were discontinued.

### 2.2. Variables

As a thirst scale, the mean thirst scores were measured for each patient using a 10-centimeter self-rating visual analog scale (VAS), from zero to ten, in which zero meant no urge to seek fluid consumption and ten meant extreme thirst. Participants were asked to record the amount of water consumed and complete questionnaires related to their liquid consumption at the beginning of each dialysis session. Interdialytic weight gain (IDWG) was also documented by measuring the patients' weight after each session and before the start of the next session using a calibrated scale.

### 2.3. Randomization and Allocation

This study used balanced 4-block randomization. For the allocation sequence, we applied for computer-generated random numbers. Medicines containing DS seeds or placebo were placed in identical numerically-coded (from 1 to 53) sealed envelopes. The patients were randomly allocated into two experimental groups: group 1 (*n* = 25) was initially treated with DS, and group 2 (*n* = 28) received a placebo initially. The groups were identical in terms of baseline characteristics and comorbidities. Daru Pajooh Jaber Company (Tabriz, Iran) supplied the treatment drugs and placebos.

### 2.4. Plant Preparation and Experimental Groups

The seeds of *Descurainia sophia* were obtained from the Tehran botanical market and identified and authenticated in Herbarium of Faculty of Pharmacy, Alborz University of Medical Sciences. According to the policy of the herbarium, a specific number as “market sample code” is given for such a sample, and the sample is kept for occasional checking during the study (market sample code: Do1-032). A hydroalcoholic extract of DS was prepared as previously described [34]. Firstly, the seeds were dried and pulverized into a fine powder using a laboratory pestle and mortar. The powder was dissolved in 96% ethyl alcohol (22 g per 21 mL) and agitated on an orbital shaker for 24 hours. The extract was condensed using a rotary-evaporator device to allow for ethanol removal. The extract was converted into powder at 60°C for 24 hours. The drug and the placebo were identical in terms of flavor and color.

Each patient in group 1 received 2 grams of DS extract every day before breakfast for six weeks, and then they underwent four weeks of washout followed by six weeks of placebo treatment. In group 2, the patients initially received a placebo for six weeks and four weeks of washout subsequently, followed by six weeks of treatment with 2 grams of DS extract every day before breakfast. The DS powder used in the treatment arm consisted of 2 grams of DS powder plus 0.5 grams of brown sugar. The placebo was prepared by combining 2 g starch powder and 0.5 g brown sugar. DS powder and placebo were prepared as sachets, and all patients were instructed to treat them as mixed syrups. The participants were told to use the sachets with 100 CCs of water. The study's outcome measures were assessed at the beginning, before washout, after washout, and at the end of the study. Patients in both also received that standard of care given to hemodialysis patients.

Patients, clinical investigators, laboratory analysts, and health care staff were all blinded to the study details regarding the treatment with DS or assignment of the matching placebos during the study. A single nurse, unaware of the contents of sachets, dispensed labeled drugs between patients and collected all the basic results throughout the research. The primary outcomes of the current study were variations in laboratory biochemical indices, oxidation factors, and thirst score in HD patients.

Blood samples were drawn in four steps: at the start of the study (1st measurement), prewashout (2nd measurement), postwashout (3rd measurement), and at the end of the study (measure 4).  Figure 1 provides a simplified study workflow.

### 2.5. Assessment of Biochemical Indices

The serum levels of calcium, cholesterol, and triglycerides were tested using colorimetric methods on a calibrated automatic blood biochemistry analyzer (ELITechGroup Clinical Systems, France). A closed electrolyte analyzer system tested potassium and sodium serum levels (Cardium, China). Malondialdehyde (MDA) as one of the final products of lipid peroxidation and as a marker of oxidative stress and the antioxidant status was measured in our study to assess the status of lipid peroxidation. MDA concentration was determined by a colorimetric assay kit and according to the manufacturer's instructions (Northwest Life Science Specialties). Total antioxidant capacity (TAC) levels were also measured based on the manufacturer's instructions (Zellbio and Axis-Shield).

### 2.6. Sample Size

As this is the first study determined to show the effects of *Descurainia sophia* on oxidative stress markers and thirst alleviation in hemodialysis patients, according to the optimal sample size estimation for a pilot randomized trial approach, a sample size of 60 participants is sufficient enough to detect a clinically significant effect size of 30% between groups, using a two-sided *Z*-test of the difference between proportions with 90% power and a 5% significance level [35].

### 2.7. Statistical Analysis

The departure from the normality assumption was assessed by the Kolmogorov–Smirnov test. A mean ± standard deviation (SD) was used for presenting the data with a normal distribution. Categorical data are presented as frequency and percentage. To evaluate the intervention effect, taking into consideration the cross-over clinical trial design of the study, a linear mixed random effect model and repeated measures analysis of variance were undertaken. Analyses were performed using STATA 13 MP. A *p* < 0.05 was considered statistically significant.

## 3. Results

A total of 53 patients were recruited for the study, including 23 (43.4%) males and 30 (56.6%) females. The mean and SD of the participants' age was 54 ± 13 years. Baseline values and alterations in thirst scores, serum calcium, potassium, triglycerides, cholesterol, total antioxidants, and weight of the patients at the end of each treatment period in the cross-over trial are shown in Table 1. The CONSORT flowchart of this study is depicted in Figure 2.

Administration of DS has significantly reduced the thirst sensation in patients on maintenance hemodialysis. The thirst score in the drug group was 0.38 units on average lower than the placebo group's (Table 2). Moreover, the results demonstrated that the interaction effect treatment × effect (carry-over effect) was not significant (estimate = 0.12, *p* value = 0.11). The effect of period was also not significant (estimate = 0.001, *p* value = 0.970). Patients in group 1 had higher mean thirst scores before DS administration. Treatment with DS led to a significant decrease in thirst VAS score (*p*=0.0001). Conversely, switching from DS to placebo in group 2 increased perceived thirst (*p* < 0.0001). The drug group's mean thirst score was lower in both periods (Figure 3).

The results of biochemical assays in Table 2 demonstrated no significant changes in serum levels of potassium and calcium throughout the study (*p* value = 0.97, *p* value = 0.49, respectively). However, the results showed that after adjusting the analysis for the baseline variables, the mean cholesterol levels in the DS group were 9.19 units lower than the mean cholesterol in the placebo group on average (*p* value <0.046). A downward trend for triglyceride concentration was observed for those receiving DS, as the mean serum triglyceride levels in the DS group were, on average, 23.93 units lower than the mean serum triglyceride level in the placebo group (*p* value <0.003). Furthermore, the results showed a significant decrease (317 units on average) in MDA levels after DS treatment (*p* value <0.001), and it seems that this beneficial effect of DS lasts even after the conversion of the regimen from DS to placebo. These results align with the measurements of TAC levels, which have an increasing trend during the study period (0.98 units on average) (*p* value = 0.001).

Results showed that cholesterol, triglycerides, Na, OXLDL, and ANT levels were significantly different between pre and post-DS in Group I. However, in Group II, the cholesterol, triglycerides, OXLDL, and ANT levels were significantly different between pre- and post-DS (Table 3). Compared to placebo, higher mean levels of calcium (*p*=0.007) and lower levels of Na (*p* < 0.001) and ANT (*p* < 0.001) were reported in Group I. However, lower OXLDL (*p*=0.005) and higher ANT (*p* < 0.001) were observed in DS compared to placebo for Group II (Table 4). The mean changes in potassium, calcium, Na, and OXLDL significantly differed between Group I and Group II; while, mean changes did not remarkably differ between two groups in cholestrol, triglycerides, and ANT (Table 5).

There was a significant decreasing trend in patients' weight after each dialysis session and between each step (*p* value <0.001). Treatment with *Descurainia sophia* was accompanied by a significant decrease in each group, but the subjects' weight was statistically similar between the two groups (*p* value = 0.539 for comparison of group 1 and group 2) (Figure 4).

No significant adverse effects were noted following treatment with DS syrup administration, except in one patient who reported nausea and vomiting. The use of a placebo did not result in any noticeable complications.

## 4. Discussion

The findings of this study demonstrated a significant reduction in thirst score, cholesterol levels, triglycerides, and malondialdehyde after four weeks of administration of DS seeds in hemodialysis patients compared to the placebo. These changes were accompanied by increased mean levels of TAC but no alterations in serum concentrations of calcium and Na+ (*p* > 0.05). To the best of our knowledge, this study is the first randomized, triple-blinded, placebo-controlled clinical trial for determining the effects of DS on systemic oxidation stress, thirst sensation, lipid profile, and serum electrolyte levels of hemodialysis patients. Previous studies have reported an elevated level of lipids in the sera of dialysis patients, which promotes atherosclerosis and is associated with excessive morbidity and mortality rates in this population [36, 37]. Similar to our findings, Mardani et al. showed that daily consumption of 8 grams of DS and 20 mg lovastatin over five months decreased the serum LDL level, but this effect was not statistically significant compared to lovastatin [38].

DS seeds contain various types of polyunsaturated fatty acids, and the lipid derivatives comprise 76.65% of the content of the extract [23, 39]. A number of these fatty acids, such as linoleic acid and oleic acid, have been previously reported to reduce LDL levels [17, 18, 40–43]. Zare et al. demonstrated that certain compounds derived from DS could stop linoleic acid saturation by omega-3 fatty acid desaturases. Moreover, another study suggested that DS inhibits the HMGR gene, reducing serum LDL levels, as seen with garlic consumption [42, 44]. These findings could be linked to the decreased LDL cholesterol levels in patients receiving DS treatment.

This study also revealed sizable effects of DS on antioxidant capacity after consumption of DS for four weeks, which was represented by a significant decrease in serum MDA levels and a considerable increase in TAC. The accumulation of MDA is related to the pathogenesis of multiple cerebrovascular and cardiovascular diseases. ESRD patients are in a high oxidative and lipid peroxidation state mainly due to inflammatory responses in these patients [45]; therefore, antioxidant supplementations seem to be of use in counteracting the oxidative state. Although despite substantial attempts, there is no definitive drug to address this complication [46, 47]. Following our findings, Moshaie-Nezhad et al. illustrated the beneficial effect of DS on hepatic oxidative damage in mice and the inverse dose-dependent relation between DS extract and MDA serum levels [34]. Consistent with our findings, the authors of a recent study used the TEAC (Trolox equivalent antioxidant capacity) assay as a surrogate marker for antioxidant capacity in vitro and demonstrated the high value of esterified phenolic fractions in DS. Their results alluded to the possible role of DS in modulating free radical scavenging [48].

As mentioned earlier, DS seed contains flavonoids capable of inhibiting lipid oxidation [49]. Safari and Sheikh reported that some flavonoids in DS, such as Morin and quercetin, protect against lipid oxidation stress [50]. In this regard, Mirzaei et al. also demonstrated the ability of the antioxidant properties of DS with similar results to our own [21]. Previous investigations considered that polyphenolic components could diminish LDL oxidation [51, 52]; they suggested that high phenol compounds in DS could explain this phenomenon [21]. These findings can steer future studies toward isolating the constructive components of DS for clinical and therapeutic utilization. Flavonoids and lignans, isolated from the extract of DS seeds, have been reported to have potent anti-inflammatory effects by inhibiting NO synthesis [22–24, 39, 43].

The inflammatory state of renal failure is considered a novel risk factor for atherosclerosis. To this end, several herbal and chemical drugs have been studied to alleviate inflammatory states with conflicting results in humans and animals [42, 46, 53–55]. Due to the general interest of the public in traditional medicine and their high compliance in this manner, numerous studies have been conducted to evaluate the efficacy of their potentially beneficial properties on inflammatory markers and lipid profiles.

Chronic volume overload in dialysis patients is associated with increased mortality and morbidity risk. Although controlling salt and water intake in these patients is important, it is impeded by patient non-compliance due to their extensive thirst. Treatment of excessive thirst in renal and heart failure patients is challenging, with no effective regimen at the moment [5, 32, 56, 57]. DS held therapeutic potential in this regard and was purportedly used to alleviate thirst in TPM [17, 58]. We, therefore, used a reliable VAS [5] to quantify and assess thirst in the hemodialysis patients in each arm. Our results demonstrated that DS effectively alleviated thirst sensation scores in this study (*p* < 0.05).

Hyperkalemia is a common finding in hemodialysis patients, significantly contributing to these patients' morbidity and mortality. The potassium content of DS is about 400 mg/kg, which is considerably higher than other medicinal herbs [59]. Despite this high potassium load, our results showed that the serum potassium levels were unchanged in hemodialysis patients receiving DS compared to the placebo. The results didn't show significant effects of DS on serum sodium levels after the intervention, although the sodium content of this herb is low [59].

It is important to note that no significant adverse effects or undesirable consequences were observed in this study. Although DS is established as a safe TPM, headaches are reportedly a frequent side effect of DS seed consumption [29, 60]. Previous works generally consider controlled use of DS derivatives safe (LD_50_ of up to 2500 mg/kg b. wt.) [28, 61].

Although the small sample size in the current study precludes definitive conclusions, the results suggest that DS consumption is beneficial through regulating electrolytes, reducing cardiovascular risk factors, augmenting antioxidant factors in dialysis patients, and reducing thirst sensation. Further pharmacokinetics, pharmacodynamics, and molecular studies that evaluate the possible downstream molecular mechanisms of components responsible for DS biological effects are recommended to verify the contradicting results. Determining potassium concentrations in the stool of the patients after DS intake may also provide insight into higher tolerance to hyperkalemia after consuming the herb in hemodialysis patients with impaired potassium clearance. Further studies are needed to clarify the effects of DS in larger populations. Furthermore, extended follow-up of intervened patients is required to evaluate the long-term effects of DS prescription.

## 5. Conclusions

Overall, this trial supports the notion that DS has pharmacological advantages as a cheap and accessible drug in hemodialysis patients and could lower cardiovascular risks. Considering that there is no conventional drug to modulate thirst sensation in this population, this study presents promising results to be further investigated in future studies.

## Figures and Tables

**Figure 1:** Study design and workflow (cross-over clinical trial).

**Figure 2:** The CONSORT flowchart.

**Figure 3:** Comparative box plot of mean thirst scores before and after the intervention.

**Figure 4:** Comparative box plot of patient's weight in four steps of the study. Group 1 (*n* = 25) and group 2 (*n* = 28). The steps are the patient's weight before and after dialysis at the first and second month of treatment.

**Table 1:** Baseline values and changes after four weeks of treatment with DS in thirst scores, serum calcium, sodium, potassium, triglycerides, cholesterol, and total antioxidant capacity of the patients at the end of each treatment period in the crossover trial.

Variables	Group I (*DS administration followed by placebo)*			Group II (*placebo followed by DS administration)*		
	Baseline	Change after six weeks	*p* value	Baseline	Change after six weeks	*p* value
Thirst VAS	9.7 ± 0.2	6.6 ± 1.6	0.0001 ^*∗∗*^	9.6 ± 0.3	9.4 ± 0.4	0.038 ^*∗*^
Calcium (mg/dl)	8.2 ± 0.6	7.8 ± 0.77	0.046 ^*∗*^	7.8 ± 0.6	8.5 ± 0.6	0.0001 ^*∗∗*^
Sodium (mEq/L)	136 ± 4.2	136 ± 2.1	0.99	145 ± 6.4	136 ± 3.5	0.0001 ^*∗*^ ^*∗*^
Potassium (mEq/L)	5.7 ± 0.89	5.5 ± 0.61	0.34	5.6 ± 0.85	5.8 ± 0.89	0.39
Triglycerides (mg/dl)	193 ± 38	187 ± 43	0.60	210 ± 43	200 ± 39	0.36
Cholesterol (mg/dl)	155 ± 49	149 ± 39	0.63	162 ± 46	147 ± 45	0.22
Malondialdehyde (*μ*mol/l)	1451 ± 748	1359 ± 684	0.65	1646 ± 690	1170 ± 622	0.009 ^*∗∗*^
TAC (mmol trolox equiv./L)	0.79 ± 0.53	1.08 ± 0.76	0.12	0.8 ± 0.51	1.0 ± 0.4	0.10

DS, *Descurainia sophia*; TAC, total antioxidant capacity.  ^*∗*^*p* value of <0.05 is considered significant.  ^*∗∗*^*p* value of <0.01 is considered highly significant.

**Table 2:** Effects of DS on oxidative stress markers and thirst alleviation using the coefficient estimation in linear mixed effect carry-over with random intercept and interaction.

	Effect	Estimate	SE	DF	*T* value	*p* value
Thirst score	Intercept	2.21	0.06	51	34.95	<0.001
	D.S. treatment	−0.38	0.11	1452	−3.30	0.001
	Time	0.001	0.04	1452	0.03	0.970
	Treatment*∗*time	0.12	0.08	1452	1.59	0.110

Potassium (mEq/L)	Intercept	4.39	0.39	96	11.33	<0.001
	D.S. treatment	>0.01	0.07	0.95	0.03	0.979
	Time	−0.03	0.07	95	−0.35	0.727
	Carry-over	0.23	0.11	96	2.07	0.041
	Baseline	0.128	0.05	95	2.51	0.014

Cholesterol (mg/dl)	Intercept	83.14	16.67	98	4.99	<0.001
	D.S. treatment	−9.19	4.55	95	2.02	0.046
	Time	14.51	4.59	95	3.16	0.002
	Carry-over	0.362	6.54	98	0.06	0.956
	Baseline	0.041	0.057	95	0.76	0.467

Calcium (mg/dl)	Intercept	3.15	0.89	96	3.53	0.001
	D.S. treatment	−0.20	0.29	58	0.70	0.490
	Time	0.39	0.29	58	1.38	0.172
	Carry-over	−0.10	0.30	96	−0.35	0.731
	Baseline	0.56	0.08	58	7.36	<0.001

Triglycerides (mg/dl)	Intercept	111.18	23.77	98	4.68	<0.001
	D.S. treatment	−23.93	7.82	97	3.06	0.003
	Time	−15.82	7.81	97	−2.02	0.056
	Carry-over	−6.39	10.37	98	−0.62	0.539
	Baseline	0.055	0.036	97	1.53	0.129

Sodium (mEq/L)	Intercept	119.88	7.94	96	15.10	<0.001
	D.S. treatment	0.11	1.02	69	0.11	0.913
	Time	0.29	1.04	69	0.28	0.779
	Carry-over	3.48	1.12	96	3.12	0.002
	Baseline	0.075	0.05	69	1.39	0.168

Malondialdehyde (*μ*mol/L)	Intercept	608.21	231.21	98	2.63	0.010
	D.S. treatment	−316.99	81.16	93	3.91	<0.001
	Time	−73.68	82.95	93	−0.089	0.377
	Carry-over	−137.95	96.43	98	−1.43	0.156
	Baseline	0.19	0.06	93	3.22	0.002

TAC (mmol trolox equiv./L)	Intercept	2.46	0.18	98	13.83	<0.001
	D.S. treatment	0.98	0.08	95	−12.91	<0.001
	Time	0.03	0.08	95	0.43	0.667
	Carry-over	−0.12	0.07	98	−1.72	0.089
	Baseline	0.25	0.05	95	4.61	<0.001

DS, *Descurainia sophia*; SE, standard error; DF, degrees of freedom; TAC, total antioxidant capacity.

**Table 3:** The comparison of outcomes between pre- and post-DS or placebo for different study groups and period.

	Group I (DS administration followed by placebo)				Group II (placebo followed by DS administration)			
	Study groups	Pre	Post	*p* value ^*∗*^	Study groups	Pre	Post	*p* value
Thirst score	DS	8.5 ± 0.9	7.5 ± 0.86	0.004	Placebo	8.3 ± 0.86	8.0 ± 0.67	0.14
	Placebo	7.9 ± 0.89	8.1 ± 0.76	0.57	DS	8.1 ± 0.98	6.4 ± 0.54	<0.001

Potassium (mEq/L)	DS	5.59 ± 0.85	5.54 ± 0.64	0.670	Placebo	5.69 ± 0.90	5.32 ± 0.62	0.119
	Placebo	5.50 ± 0.62	5.51 ± 0.54	0.920	DS	5.84 ± 0.89	5.32 ± 0.61	0.007

Cholesterol (mg/dl)	DS	162.37 ± 46.70	114.29 ± 31.39	<0.001	Placebo	154.83 ± 49.25	123.34 ± 35.09	0.006
	Placebo	149.59 ± 38.92	137.64 ± 39.03	0.091	DS	200.30 ± 102.95	108.00 ± 33.76	0.101

Calcium (mg/dl)	DS	7.85 ± 0.60	7.95 ± 0.78	0.406	Placebo	8.13 ± 0.60	8.37 ± 0.70	0.058
	Placebo	7.85 ± 0.78	8.48 ± 0.80	<0.001	DS	8.50 ± 0.00	8.38 ± 0.85	—

Triglycerides (mg/dl)	DS	209.94 ± 129.32	117.96 ± 35.21	<0.001	Placebo	193.40 ± 94.88	147.37 ± 89.25	0.059
	Placebo	187.01 ± 104.85	124.81 ± 71.49	<0.001	DS	200.30 ± 102.95	108.00 ± 33.76	<0.001

Na	DS	144.78 ± 6.48	138.07 ± 3.68	<0.001	Placebo	135.83 ± 4.24	134.03 ± 3.63	0.073
	Placebo	136.26 ± 2.35	137.84 ± 3.01	<0.001	DS	135.67 ± 3.51	134.10 ± 3.27	0.667

OXLDL	DS	1645.96 ± 690.66	882.44 ± 380.83	<0.001	Placebo	1451.03 ± 748.13	1301.08 ± 875.57	0.466
	Placebo	1359.45 ± 683.99	1071.63 ± 631.66	0.004	DS	1170.22 ± 622.63	846.17 ± 429.22	0.021

ANT	DS	0.80 ± 0.52	1.47 ± 0.71	<0.001	Placebo	0.79 ± 0.54	0.62 ± 0.21	0.087
	Placebo	1.08 ± 0.77	0.60 ± 0.20	<0.001	DS	0.99 ± 0.41	1.68 ± 0.55	<0.001

Malondialdehyde (*μ*mol/L)	DS	1709 ± 720	882 ± 380	<0.001	Placebo	1695 ± 743	758 ± 295	<0.001
	Placebo	927 ± 351	786 ± 350	0.009	DS	851 ± 334	846 ± 429	0.91

TAC (mmol trolox equiv./L)	DS	0.77 ± 0.5	0.91 ± 0.67	0.003	Placebo	0.8 ± 0.55	0.89 ± 0.6	0.24
	Placebo	1.07 ± 0.76	0.96 ± 0.58	0.32	DS	1.15 ± 0.8	0.85 ± 0.5	0.09

Values are expressed as means ± SD; the drug-placebo group took the drug at first, while the placebo-DS group received a placebo following DS.  ^*∗*^The paired *t*-test was used to compare the outcomes change before and after the DS or placebo in each study group. DS, *Descurainia sophia*.

**Table 4:** The comparison of outcomes between placebo and treatment for different sequence.

	Group I (DS administration followed by placebo)				Group II (placebo followed by DS administration)			
	Study groups	DS	Placebo	*p* value ^*∗*^	Study groups	Placebo	DS	*p* value
Thirst score	DS-placebo	6.6 ± .76	9.8 ± 0.93	<0.001	Placebo-DS	9.7 ± 0.78	8.2 ± 0.76	<0.001
Potassium (mEq/L)	DS-placebo	5.57 ± 0.75	5.50 ± 0.58	0.418	Placebo-DS	5.51 ± 0.79	5.59 ± 0.80	0.586
Cholesterol (mg/dl)	DS-placebo	138.33 ± 46.41	143.65 ± 39.29	0.302	Placebo-DS	139.36 ± 45.38	137.48 ± 43.90	0.819
Calcium (mg/dl)	DS-placebo	8.34 ± 0.46	8.23 ± 0.39	0.391	Placebo-DS	8.25 ± 0.66	8.39 ± 0.83	0.408
Triglycerides (mg/dl)	DS-placebo	163.95 ± 105.11	155.91 ± 94.70	0.502	Placebo-DS	170.38 ± 94.23	154.15 ± 89.08	0.334
Na	DS-placebo	141.43 ± 6.24	137.05 ± 2.81	<0.001	Placebo-DS	134.93 ± 4.02	134.25 ± 3.26	0.414
OXLDL	DS-placebo	1266.95 ± 675.84	1215.54 ± 671.68	0.525	Placebo-DS	1377.33 ± 809.73	1011.04 ± 556.21	0.005
ANT	DS-placebo	1.14 ± 0.70	0.84 ± 0.61	<0.001	Placebo-DS	0.71 ± 0.42	1.34 ± 0.59	<0.001
Malondialdehyde (*μ*mol/L)	DS-placebo	1687 ± 402	946 ± 567	<0.001	Placebo-DS	997 ± 468	1578 ± 668	0.0005
TAC (mmol trolox equiv./L)	DS-placebo	0.97 ± 0.43	0.78 ± 0.38	0.093	Placebo-DS	0.83 ± 0.32	1.06 ± 0.49	0.046

Values are expressed as means ± SD; the drug-placebo group took the drug at first, while the placebo-DS group received a placebo following DS.  ^*∗*^The paired *t*-test was used to compare the outcomes change between DS (pre + post values) and placebo (pre + post values) in each study group. DS, *Descurainia sophia*.

**Table 5:** The comparison of mean changes in outcome between groups.

Group I (DS administration followed by placebo) vs. Group II (placebo followed by DS administration)				
	Study groups	DS-placebo	Placebo-DS	*p* value*∗*
Thirst score	Average (diff DS-diff placebo) vs. average (diff placebo-diff DS)	−2.4 ± 0.87	−1.9 ± 0.69	0.023
Potassium (mEq/L)	Average (diff DS-diff placebo) vs. average (diff placebo-diff DS)	−0.02 ± 0.89	−0.80 ± 1.73	0.001
Cholesterol (mg/dl)	Average (diff DS-diff placebo) vs. average (diff placebo-diff DS)	−31.00 ± 57.05	−27.48 ± 61.46	0.697
Calcium (mg/dl)	Average (diff DS-diff placebo) vs. average (diff placebo-diff DS)	0.69 ± 2.06	4.03 ± 4.16	<0.001
Triglycerides (mg/dl)	Average (diff DS-diff placebo) vs. average (diff placebo-diff DS)	−77.09 ± 121.52	−69.17 ± 119.32	0.671
Na	Average (diff DS-diff placebo) vs. average (diff placebo-diff DS)	−2.53 ± 6.96	57.17 ± 67.92	<0.001
OXLDL	Average (diff DS-diff placebo) vs. average (diff placebo-diff DS)	−531.97 ± 796.47	−267.39 ± 901.84	0.040
ANT	Average (diff DS-diff placebo) vs. average (diff placebo-diff DS)	0.10 ± 0.91	0.24 ± 0.67	0.287

Values are expressed as means ± SD; the drug-placebo group took the drug at first, while the placebo-DS group received a placebo following DS. *∗*The independent *t*-test was used to compare the mean change between study groups. DS, *Descurainia sophia*.

## Data Availability

The data used to support the findings of this study are available from the corresponding author upon request.
